The article "Magnitude and associated factors of mortality among patients admitted with COVID-19 in Addis Ababa, Ethiopia" was retracted in 2024. Reasons: duplicate publication; overlap with earlier publications.

# Magnitude and associated factors of mortality among patients admitted with COVID-19 in Addis Ababa, Ethiopia

**DOI:** 10.1371/journal.pgph.0000420

**Published:** 2023-08-17

**Authors:** Genanew Kassie Getahun, Amare Dinku, Dube Jara, Tewodros Shitemaw, Zelalem Negash

**Affiliations:** 1 Menelik II Medical and Health Science College, Kotebe Metropolitan University, Addis Ababa, Ethiopia; 2 Yanet Health College, Addis Ababa, Ethiopia; 3 Debre Markos University, Debre Markos, Ethiopia; 4 Yekatit 12 Medical College, Addis Ababa, Ethiopia; Epicentre MSF, SWITZERLAND

## Abstract

The COVID-19 pandemic continues to grow around the world and has caused enormous mortality and morbidity. The severity and mortality of coronavirus disease are associated with various comorbidities. The infection fatality rate was reported to be inconsistent with different studies. Therefore, the aim of this study was to assess the magnitude and factors associated with mortality among patients admitted to Eka Kotebe General Hospital, Addis Ababa, Ethiopia. An institutional-based cross-sectional study was conducted at Eka Kotebe General Hospital among patients who were admitted for COVID-19 from January 15, 2021, to June 30, 2021. A total of 393 records of patients were selected by simple random sampling. Data was extracted from compiled data forms where available information was already tabulated. Data was entered and analyzed using SPSS version 25. The determinant factors associated with mortality among COVID-19 patients were identified using bivariate and multivariable logistic regression analysis. A statistical association was declared with multivariable logistic regression using a 95% confidence interval and a P-value of less than 0.05. The proportion of COVID-19 mortality among patients admitted to Eka Kotebe General Hospital was 8.1% (95% CI (5.4–10.8%)). Age >50 years [AOR = 7.91; 95% CI (2.34–25.70)], being male [AOR = 2.09; 95% CI (1.20–3.65)], having diabetes mellitus [AOR = 2.64; 95% CI (1.30–5.35)], having hypertension [AOR = 2.67; 95% CI (1.22–5.88)] and having chronic kidney disease [AOR = 12.04; 95% CI (4.03–14.22)] were determinant factors of COVID-19 mortality. The current study findings revealed that COVID-19 mortality was high among hospitalized COVID-19 patients. Furthermore, age, gender, diabetes mellitus, hypertension, and chronic kidney disease were discovered to be independent predictors of COVID-19 mortality. Therefore, older COVID-19 patients and those with established comorbidities such as hypertension, diabetes, and end-stage renal disease should receive comprehensive preventative efforts, including vaccination.

## Introduction

There has been a significant loss of human life as a result of the novel coronavirus illness 2019 (COVID-19), which is still spreading throughout the world and causing tremendous mortality and morbidity [1]. This has created an unmatched challenge for the provision of public health services [2]. Those who have had preexisting medical illnesses in the past or who are currently suffering from medical disorders are seriously affected [3].

African countries (with a median age of less than 20 years) have registered a lower number of severe COVID-19 cases and deaths than Europe and the United States (median age > 38 years), despite a number of underlying factors like malnutrition, risky livelihoods, cultural factors, economic factors, and overcrowding within urban settlements [4, 5]. A lower case fatality rate was also observed in Africa when compared to the Americas and Europe; however, it was more or less comparable to Asia [6].

Excess mortality measures have been used to assess the impact of COVID-19 pandemics on public health, particularly when there are concerns about the under-counting of deaths that are directly related to a particular event or cause [7]. The disruption of societal and health systems, deaths from other causes, and the long-term health impact of COVID-19 in Sub-Saharan Africa are uncertain, especially given the region’s poor testing capacity [8, 9].

Ethiopia’s Federal Ministry of Health reported the first COVID-19 case in Addis Ababa on March 13, 2020, and Ethiopia is one of the most severely affected African countries, suffering terrible economic and medical hardships [10]. A report by February 2022 indicates that Ethiopia is seeing a modest decline in COVID-19 infections. On average, 121 new illnesses were recorded each day, that is much lower than the highest daily average ever recorded since the outbreak started. Since the start of the pandemic, there have been 468,345 illnesses and 7,438 deaths attributed to the coronavirus throughout the nation [11].

It is well established that a number of comorbidities are connected to both the severity and mortality of coronavirus disease [12]. Findings from a prospective cohort study showed that hypertension (23.5%), obesity (19.6%), and osteoarthritis (14.9%) were the most common, whereas chronic viral hepatitis type C (0.6%), type B (0.3%), and HIV (0.3%) were the least common [13]. Moreover, patients with a history of cardiovascular illness, chronic lung disease, or diabetes had the worst prognosis and were more likely to experience deteriorating outcomes like acute respiratory distress syndrome (ARDS) and pneumonia [13, 14]. It was associated with a substantial risk of mortality and severe morbidity in cancer patients [15]. When comparing patients with COVID-19 who had been hospitalized without comorbidity, the risk of mortality was lower in COVID-19 patients admitted with diabetes mellitus, hypertension, or cardiovascular disease (CVD) [16].

COVID-19 is currently a global discussion topic in the media and with the public. The outbreak has been declared an emergency, with the community facing an increased risk of infection. To our knowledge, few studies have been undertaken in Africa at a time when the pandemic appears to be different from that of other continents in terms of virus dissemination speed and death toll. As a result, the purpose of this research was to look at the magnitude of mortality and its associated factors among COVID-19 patients admitted to the Eka Kotebe General Hospital treatment center, Addis Ababa, Ethiopia.

## Methods

### Time and place of study

The study was conducted in Addis Ababa, Ethiopia. Addis Ababa city has 11 sub-cities. The city administration had an estimated total population of 5,005,524, where 7.16% were children under the age of five [17]. Eka Kotebe General Hospital (treatment center) is one of the seven federal government hospitals located in Addis Ababa. The hospital serves as a COVID-19 referral treatment center with more than 600 beds for COVID-19 patients and over 400 clinical staff. The hospital underwent extensive renovations and was converted into a COVID-19 treatment facility in September of 2019 where COVID-19 patients were isolated and treated as a result of the COVID-19 outbreak. The study was conducted between January 15, 2021, and June 30, 2021.

### Study design and population

An institutional-based cross-sectional study was conducted with randomly selected patients infected and confirmed by PCR tests of COVID-19 and admitted to Eka Kotebe General Hospital between January 15 and June 30, 2021. The total number of patients admitted with COVID-19 during the study period was 4,876.

### Inclusion and exclusion criteria

#### Inclusion

Patients who had been infected with COVID-19 and were admitted either to emergency, ICU, or critical care wards and who were more than 18 years old were included.

#### Exclusion

Patients who had incomplete documentation were excluded.

### Sample size and sampling procedure

The sample size was calculated using a single population proportion formula, considering the prevalence of COVID-19 mortality to be 50% to have the largest sample size with a 95% confidence level and a 5% margin of error. Finally, adding a non-response rate of 10%, it was 422.

With a simple random sampling technique, respondents were selected using the total number of admitted patients as a source population and their medical record numbers as a sampling frame. Subsequently, lottery methods were applied to select study participants randomly. In general, using the patient registry as a source document, random patients were selected in Eka Kotebe general hospital and admitted as COVID-19 patients.

### Study variables

#### Dependent variables

COVID-19 related mortality (yes or no) between January 15, to June 30, 2021.

#### Independent variables

Sociodemographic factors

Clinical factors

Comorbidities

Pregnancy and childbearing

Malnutrition and micronutrient deficiency

#### Data collection procedures and quality control

Data was gathered from hospital documents using checklists in various wards, such as the ICU, critical care units, and emergency rooms. Computer-based registration formats were used to collect the data. To ensure the quality of the data, two professional nurses were recruited, and training was given on the data collection procedures, purposes of the study, categorization, and coding of the data. Every day, the activities were reviewed and checked for completeness and relevance by the principal investigators. Finally, the collected data was transferred to a secured area.

### Operational definition

#### Co-morbid disease

A chronic disease or group of chronic diseases that are present concurrently in COVID-19-infected patients.

#### Clients or patients

COVID-19-hospitalized individuals or COVID-19-infected individuals admitted to Eka Kotebe General Hospital for medical treatment.

#### Mortality

The number of deaths out of all admitted individuals infected by COVID-19 in Eka Kotebe General Hospital.

#### Data processing and analysis

Data entry was made using Epi Data version 3.1 and exported to SPSS version 25, for further analysis. Frequencies, proportions, and summary statistics were used to describe the study population in relation to relevant variables. Basic assumptions for binary logistic regression were done and model fitness has been checked before running multiple logistic regression analysis. Initially, binary logistic regression analysis was employed to analyze the relationship between independent variables and COVID-19 related mortality, along with the odds ratio and its 95% confidence interval. The variables with a p-value less than 0.25 were then incorporated into a multivariable logistic regression model, as suggested by Hosmer and Lemeshow [18]. In addition, each morbidity was assessed at binary logistic regression for being a candidate of multivariable logistic regression analysis and for being an independent driver of COVID-19 related mortality in the final model. Variables with a p-value of less than 0.05 were used to declare their statistical significance. The result was finally presented using text, tables, and charts based on the characteristics of the data.

### Ethical consideration

Ethical approval was obtained from Yanet College’s research and ethics board. A permission letter was secured from the institutional review board of Eka Kotebe General Hospital. Data was collected after receiving informed written consent from each study participant. Confidentiality was ensured by concealing the patient profile’s name and any specific characteristics in favor of a code and medical registration number.

## Results

### Demographic characteristics of respondents

Out of a total of 422 patients and their respective records, 393 patients and records with complete responses were chosen, yielding a response rate of 93.1%. Of the total participants, 233 (59.3%) were under the age of 50. In terms of gender, nearly two-thirds of the 252 (64.1%) participants were males, with a male-to-female ratio of more than 3:2.

In addition, 141, or 35.9%, of the male participants in this study were under the age of 50, while the remaining 111, or 28.2%, were 50 or older. In contrast, 49 (12.5%) and 92 (23.4%) of the study’s female participants were, respectively, under 50 and over 50.

### The magnitude of COVID-19 mortality

Of the total COVID-19 patients and records evaluated, 32 (8.1%; 95% CI: (5.4–10.8%)) died as a result of COVID-19-related illnesses (Fig 1).

**Fig 1:** COVID-19 mortality among patients admitted to the COVID treatment center in Eka Kotebe General Hospital, Addis Ababa, Ethiopia, 2021 (n = 393).

Furthermore, a majority of the study participants (275, or 70%) had a co-morbidity, with hypertension and other cardiovascular disorders being the most prevalent (103, or 26.2%), whereas cancer and malnutrition-related comorbidities were the least common, at 12 (3.1%) and 9, (2.3%), respectively. Records of patients were also examined in order to categorize them based on the sorts of co-morbidities they had at the time of diagnosis (Table 1).

**Table 1:** Medical conditions associated with COVID-19 among patients admitted to the COVID treatment center at Eka Kotebe General Hospital, Addis Ababa, Ethiopia, 2021 (n = 393).

Characteristics	Frequency	Percentage
Admission diagnosis		
Tuberculosis	63	16.0
HIV/AIDS	47	12.0
Cancer (All types)	12	3.1
Hypertension	103	26.2
Diabetes mellitus	82	20.9
Chronic heart disease	31	7.9
Chronic liver disease	13	3.3
Chronic kidney disease	70	17.8
Pregnancy and child birth	25	6.4
Malnutrition	9	2.3
GIT related disease	67	17.0
Skin and musculoskeletal disorder	40	10.2
Psychiatry & nervous system disorder	45	11.5
Others	22	5.6
COVID-19 associated with another comorbidity		
Yes	275	70
No	118	30

### Factors associated with COVID-19 mortality

A binary logistic regression analysis was conducted to identify the presence of the association between COVID-19 mortality and different independent variables. In the bivariate logistic regression analysis, variables that scored a p-value of less than 0.25 were selected as candidate variables for the multivariable logistic regression analysis; accordingly, age, sex, COVID-19 associated with HIV/AIDS, DM, HTN, CHD, CKD, malnutrition, micronutrient deficiency, and GIT-related disease were found to be associated with COVID-19 mortality.

Finally, the selected variables were entered into a multivariable logistic regression analysis. As a result, respondents aged 50 and above [AOR = 7.91, 95% CI: 2.34–25.69]; being male [AOR = 2.09, 95% CI: 1.20–3.65); having diabetes mellitus [AOR = 2.67, 95% CI: 1.22–5.88); and having chronic kidney disease [AOR = 12.04, 95% CI: 4.03–14.22] had a statistically significant association with COVID-19 mortality (Table 2).

**Table 2:** Risk factors for death in COVID-19 patients admitted to Eka Kotebe Hospital in Addis Ababa, Ethiopia, in 2021 (n = 393).

Variables	Death		COR (95% CI)	AOR (95%CI)
	Yes	No		
**Age of patients:**				
<50 years	8	245	1	1
≥50 years	24	116	6.34(2.76–14.53)	7.91(2.43–25.70) **
**Sex**				
Male	24	228	1.75(0.76–4.01)	2.09(1.20–3.65) *
Female	8	133	1	1
**HIV/AIDS and other hematologic disorders**				
Yes	13	34	6.58(2.99–14.48)	1.58(0.78–3.22)
No	19	327	1	1
**DM & other metabolic disease**				
Yes	15	67	3.87(1.84–8.14)	2.64(1.30–5.35) **
No	17	294	1	1
**HTN & vascular disease**				
Yes	16	87	3.15(1.51–6.56)	2.67(1.22–5.88) **
No	16	294	1	1
**CHD & related disease**				
Yes	7	24	3.93(1.54–10.01)	2.69(0.98–4.93)
No	25	337	1	1
**CKD & related disease**				
Yes	20	50	10.37(4.77–22.51)	12.04 (4.03–14.22)**
No	12	311	1	1
**Malnutrition and micro- nutrient deficiency**				
Yes	2	7	3.37(0.67–16.95)	2.04(0.83–4.02)
No	30	354	1	1
**Musculoskeletal and skin related disorders**				
Yes	7	34	2.22(0.85–5.77)	2.04(0.33–4.02)
No	25	327	1	1

*Indicates a p-value < 0.05, and

** shows a p-value < 0.01

## Discussion

The current study revealed that COVID-19 mortality was found to be 8.1% (95% CI: 5.4–10.8%) among patients admitted to Eka Kotebe General Hospital. The prevalence was higher than that of studies conducted in Nigeria (4.3%) [19] and Northern Ethiopia (0.8%) [14]. However, it was lower than a study finding from the Democratic Republic of Congo (32%) [20] and Indus Hospital Karachi, Pakistan (39%) [21]. The disparity could be attributable to differences in the study participants’ characteristics and the sample size employed. For instance, the findings from Pakistan and the Congo were reported from a small number of participants among critically ill patients, and the majority of the study participants in Northern Ethiopia were asymptomatic patients.

In a multivariable logistic regression analysis, age of patients, sex, co-morbidity among all admitted patients, diabetes mellitus, hypertension, and chronic kidney disease were found to be significant drivers of COVID-19 mortality.

Accordingly, people over the age of 50 had roughly eight times [AOR = 7.91, 95% CI: (2.34–25.69)] the odds of dying from COVID-19 compared to their younger counterparts. It’s consistent with study findings throughout the world [22–26]. This might be explained by the fact that older adults had higher rates of COVID-19-related hospitalization, and the majority of those admitted had underlying medical disorders that were common among older adults.

On the other hand, males had a twofold higher risk of COVID-19 death than females. The greater death risks linked with COVID-19 for males could be due to associated comorbidities such as cardiovascular illnesses, hypertension, obesity, diabetes, or biological or genetic factors, but they could also be due to flaws in the health-care system [27–30].

The current finding also revealed that COVID-19 patients with diabetes mellitus had a 2.6-times greater risk of death. This could be due to the fact that diabetes might predispose patients to adverse outcomes and is a substantial risk factor for the severity and death of COVID-19 patients. This is supported by a number of research findings [23, 31–34], which might be due to a weakened innate immune system caused by chronic hyperglycemia, an overactive cytokine response, and hypercoagulability-related clinical impairments [35].

Another conclusion from multivariate logistic regression analysis was that COVID-19 patients with hypertension were nearly three times more likely to die, implying that hypertension is a major predictor of hospital mortality. This conclusion is backed up by a number of studies [31, 36, 37]. It could be owing to the fact that older people have a higher risk of cardiovascular disease and diabetes (all well-known risk factors for mortality in critical patients) than younger people do.

Chronic kidney diseases were a strong predictor of COVID-19 mortality. A COVID-19 patient with CKD had twelve times higher odds of death. In a similar study of the European population, patients with high creatinine levels and a history of previous CKD were found to have a higher rate of in-hospital death [30, 31, 38]. This may be linked to their weakened immune systems. In addition, non-survivors of COVID-19 showed higher levels of variables linked to renal illness, such as creatinine, blood urea, neutrophil count, and D-dimer [39].

### Limitation

Hence, many patients with one or more comorbidities were represented, and different clinical treatment regimens were implemented. This might lead to differing survival outcomes. Due to the cross-sectional nature of the study that was performed, the association between various factors and COVID-19-associated mortality may not indicate a cause-and-effect relationship. Moreover, this study included only in-hospital patients who tested positive. Some people may have developed symptoms in the community but were not tested, or they may have been asymptomatic.

## Conclusion and recommendations

The results of the current study showed that the magnitude of COVID-19 mortality among hospitalized COVID-19 patients was high. Moreover, age, gender, and presence of co-morbidity among all admitted patients—including diabetes, hypertension, and chronic kidney disease were—discovered to be determinants of COVID-19 mortality. Therefore, older COVID-19 patients and those with established comorbidities such as hypertension, diabetes, and end-stage renal disease should receive comprehensive preventative efforts, including vaccination.

## Supporting information

S1 Table Binary logistic regression table. (DOCX)
